# In Silico and In Vitro Studies on the Mechanisms of Chinese Medicine Formula (Yiqi Jianpi Jiedu Formula) in the Treatment of Hepatocellular Carcinoma

**DOI:** 10.1155/2022/8669993

**Published:** 2022-10-29

**Authors:** Zhulin Wu, Jianyuan Kang, Wanjun Tan, Chunshan Wei, Li He, Xiaoyan Jiang, Lisheng Peng

**Affiliations:** ^1^The Fourth Clinical Medical College of Guangzhou University of Chinese Medicine, Shenzhen 518033, China; ^2^Shenzhen Traditional Chinese Medicine Hospital, Shenzhen 518033, China; ^3^Shenzhen Futian Center for Chronic Disease Control, Shenzhen 518033, China

## Abstract

**Objective:**

Traditional Chinese medicine (TCM) is an important part of the comprehensive treatment of hepatocellular carcinoma (HCC), and Chinese materia medica formulas with the effect of “Yiqi Jianpi” (replenishing qi and strengthening spleen) or “Jiedu” (removing toxicity) have been proved to be effective in treating HCC. However, mechanisms of these formulas in treating HCC remain unclear. In this paper, our goal is to explore the antitumor activity and its molecular mechanisms of Yiqi Jianpi Jiedu (YQJPJD) formula against HCC.

**Methods:**

The bioactive ingredients and targets of YQJPJD formula and HCC targets were screened by five Chinese materia medicas and two disease databases, respectively. The network pharmacology was utilized to construct the relationship network between YQJPJD formula and HCC, and the mechanisms were predicted by the protein-protein interaction (PPI) network, pathway enrichment analysis, bioinformatics, and molecular docking. Numerous in vitro assays were performed to verify the effect of YQJPJD formula on HCC cells, cancer-associated targets, and PI3K/Akt pathway.

**Results:**

The network relationship between YQJPJD formula and HCC suggested that YQJPJD formula mainly regulated the potential therapeutic targets of HCC by several key bioactive ingredients (e.g., quercetin, luteolin, baicalein, and wogonin). PPI network, bioinformatics, and molecular docking analyses displayed that YQJPJD formula may play an anti-HCC effect through key targets such as MAPK3, RAC1, and RHOA. Additionally, pathway analysis demonstrated that YQJPJD formula could play an anti-HCC effect via multiple pathways (e.g., PI3K-Akt and hepatitis B). Experimental results showed that YQJPJD formula could effectively inhibit the proliferation, migration, and invasion of HCC cells and promote HCC cell apoptosis in a concentration-dependent manner. Moreover, YQJPJD formula could decrease the mRNA expression of *β*-catenin, MAPK3, and RHOA and the protein expression of phosphorylated PI3K and Akt.

**Conclusion:**

YQJPJD formula mainly exerts its anti-HCC effect through multiple bioactive ingredients represented by quercetin, as well as multiple pathways and targets represented by PI3K/Akt pathway, *β*-catenin, MAPK3, and RHOA.

## 1. Introduction

The most common primary liver cancer is known to be hepatocellular carcinoma (HCC), whose risk factors include hepatitis B virus (HBV), hepatitis C virus (HCV), fatty liver disease, alcohol-related cirrhosis, and several dietary exposures [1]. HCC displays high frequency of relapse and metastasis, and the survival rate of patients with HCC is still poor in light of 2020 global cancer data statistics [2]. Limited therapeutic choices are available for patients with advanced-stage HCC, and current treatment consists of chemoembolization, molecularly targeted therapy, radiotherapy, and immune checkpoint inhibitors. Therefore, investigating the underlying mechanisms of HCC and developing drugs to treat HCC are of paramount importance. In China, traditional Chinese medicine (TCM) is an important part of the comprehensive treatment of cancer, which can run through the whole process of cancer treatment. Previous studies have shown that Chinese materia medica formulas, as one of the main intervention measures of TCM, can improve the survival quality of HCC patients, prolong the survival time, and reduce the side effects of chemoembolization [3, 4].

Chinese materia medicas have tremendous potential for the development of new drugs. Based on the theory of TCM, the compositions of Chinese materia medica formulas are diverse, and each formula can have a different name and specific TCM efficacy. Also, preceding studies have revealed that Chinese materia medica formulas with the effect of “Jianpi Jiedu” (strengthening spleen and removing toxicity) could promote the recovery of liver function and the quality of life of HCC patients [5], and “Fuzheng” (strengthens healthy qi) had a significant effect on patients with advanced HCC and could remarkably prolong the survival time of patients [6]. Nevertheless, the action mechanisms of these formulas also need to be further explained by modern medical research. Yiqi Jianpi Jiedu (YQJPJD) formula, with the effect of “Yiqi Jianpi Jiedu” (replenishing qi, strengthening spleen, and removing toxicity), is currently being studied in our laboratory, and YQJPJD formula contains the following 10 Chinese materia medicas: *Phyllanthus urinaria L.* (Yexiazhu in Chinese), *Astragalus membranaceus (Fisch.) Bunge* (Huangqi in Chinese), *Codonopsis pilosula (Franch.) Nannf.* (Dangshen in Chinese), *Atractylodes macrocephala Koidz.* (Baizhu in Chinese), *Poria cocos (Schw.) Wolf.* (Fuling in Chinese), *Scutellaria barbata D. Don.* (Banzhilian in Chinese), *Hedyotis diffusa Willd* (Baihuasheshecao in Chinese), *Bupleurum chinense DC.* (Chaihu in Chinese), *Paeonia lactiflora Pall.* (Baishao in Chinese), and *Glycyrrhizae Radix Et Rhizoma Praeparata Cum Melle* (Zhigancao in Chinese). Among them, *Phyllanthus urinaria L.* is a common Chinese materia medica used by our TCM team in the treatment of HCC, which demonstrated a good anti-HCC effect in both clinical and experimental studies [7, 8]. The remaining 9 Chinese materia medicas excavated by data mining are the core Chinese materia medicas for treating HCC in TCM [9], and most of these Chinese materia medicas also have good anti-HCC effects. For instance, *Astragalus membranaceus* could promote vascular normalization in tumor-derived endothelial cells of HCC by reduced expression of HIF1a [10], and the standardized extract of *Astragalus membranaceus* and *Paeonia lactiflora* caused significant inhibition of cell proliferation, migration, and invasion effect in HCC cells [11]. *Scutellaria barbata* suppressed HCC tumorigenesis in vivo by inducing ferroptosis of HCC cells [12], and *Hedyotis diffusa Willd* inhibited proliferation of HepG2 cells and potentiated the anticancer efficacy of 5-fluorouracil in treating HCC [13]. It was reported that Sijunzi decoction, a classic and famous TCM formula consisting of four components, *Codonopsis pilosula (Franch.)*, *Atractylodes macrocephala Koidz.*, *Poria cocos (Schw.)*, and *Glycyrrhizae Radix*, could inhibit gastric cancer stem cells by attenuating the transcriptional activity of *β*-catenin. However, the potential role of YQJPJD formula in cancer treatment has not been studied. Recently, the emergence of network pharmacology has innovated the traditional mode of drug research, providing new technical support for the systematic research and innovative drug development of TCM [14]. In this study, a combination of network pharmacology and experimental verification was utilized to clarify the mechanisms of YQJPJD formula in the treatment of HCC.

## 2. Material and Methods

### 2.1. Prediction of Bioactive Ingredients and Targets of YQJPJD Formula

The bioactive ingredients of YQJPJD formula were identified by using TCM System Pharmacology database (TCMSP, https://tcmsp-e.com/tcmsp.php) [15], SymMap (http://www.symmap.org) [16], Integrative Pharmacology-Based Research Platform of TCM (TCMIP, http://www.tcmip.cn/TCMIP/index.php/Home/Login/login.html) [17], Bioinformatics Analysis Tool for Molecular mechANism of TCM (BATMAN-TCM, http://bionet.ncpsb.org/batman-tcm/) [18], and HERB (http://herb.ac.cn/) [19]. The ingredients with drug-likeness (DL) ≥ 30% and oral bioavailability (OB) ≥ 18% were screened for further study [15], and the corresponding targets of bioactive ingredients of the YQJPJD formula were also obtained from the above five databases. All target names were converted to corresponding gene names through the UniProt database (https://www.uniprot.org/uniprot/).

### 2.2. Screening the Common Targets of YQJPJD Formula and HCC

The potential target genes related to HCC were acquired from MalaCards (https://www.malacards.org/) and OMIM (https://omim.org/) databases with the keyword “Hepatocellular Carcinoma”. Subsequently, the repeated target genes were removed manually, and the known target genes of HCC were screened. The Venn diagram was used to obtain the common targets of YQJPJD formula and HCC. The network of “bioactive ingredients of YQJPJD formula-common target” was established by using Cytoscape software (version 3.7.2).

### 2.3. PPI and Hub Gene Analyses

The protein-protein interaction (PPI) network of common targets was constructed by using the STRING online tool (https://string-db.org), the minimum interaction score threshold was set to be greater than 0.7, and the species was limited to “Homo sapiens.” Based on the PPI network, CytoHubba plug-in of Cytoscape software was used to determine the hub genes according to the degree algorithm.

### 2.4. Functional Enrichment Analysis for Common Targets

Gene Ontology (GO) analysis and Kyoto Encyclopedia of Genes and Genomes (KEGG) signal pathway analysis were performed on the common targets through DAVID database (https://david.ncifcrf.gov/). GO analysis is based on three types, including biological process (BP), cellular component (CC), and molecular function (MF). The top five significant items in each GO type were arranged according to false discovery rate (FDR), and the result was visualized by bar plot, and the 20 key KEGG pathways (significant enrichment) were arranged according to target count and the result was visualized by bubble chart. Data visualization is accomplished through the “bioinformatics” online platform (https://www.bioinformatics.com.cn).

### 2.5. Expression and Survival Analyses of Hub Genes

Several bioinformatics databases were utilized to analyze the expression and prognostic values of hub genes in the PPI network. The mRNA expression levels of hub genes were analyzed by UALCAN database (http://ualcan.path.uab.edu). UALCAN is a global open online tool based on The Cancer Genome Atlas (TCGA) data, which can be used to analyze gene expression levels between tumor and normal tissues [20]. Moreover, the protein expression levels of hub genes were detected using Human Protein Atlas (HPA) database (https://www.proteinatlas.org). HPA online database has abundant immunohistochemical images, which can show the expression of target protein in various tumor tissues and corresponding normal tissues [21]. In addition, the prognostic values of hub genes were evaluated by the Kaplan-Meier (KM) plotter online tool (http://www.kmplot.com) [22], which included survival and gene expression data of 364 HCC patients from the TCGA dataset. KM survival curves were performed to compare overall survival (OS) between patients with high and low hub gene expressions based on the default parameters of the KM plotter.

### 2.6. Molecular Docking Verification

In this study, molecular docking method was preliminarily utilized to validate the results of network pharmacology. Through the RCSB Protein Data Bank (PDB, http://www.rcsb.org/pdb), protein receptors of hub genes were selected according to the following criteria: (1) the structure of protein receptors was identified by X-ray diffraction, (2) X-ray resolution < 3 as the first choice, and (3) protein structures containing original ligands (e.g., inhibitors) were preferred. By using AutoDockTools1.5.6 (http://autodock.scripps.edu), the original ligands (if any), excess protein chains, and water molecules of the protein receptor were removed, then hydrogen was added to the protein receptors, and possible docking coordinates were searched. The structure (“mol2” format) of the corresponding bioactive ingredients of the target protein was obtained by TCMSP database. Subsequently, the file format of protein receptor or bioactive ingredient was converted to “PDBQT” using AutoDockTools, and molecular docking was performed using AutoDock Vina program (http://vina.scripps.edu/). Finally, the results were analyzed and visualized using PyMOL (http://www.pymol.org/) and Discovery Studio 2016.

### 2.7. In Vitro Experimental Validation

#### 2.7.1. Preparation and HPLC Analysis of YQJPJD Formula Aqueous Extract

To prepare the aqueous extract of YQJPJD formula, 30 g Phyllanthus urinaria L. (Lot no. 201001101), 30 g Astragalus membranaceus (Fisch.) Bunge (Lot no. 200900341), 15 g Codonopsis pilosula (Franch.) Nannf. (Lot no. 201001131), 15 g Atractylodes macrocephala Koidz. (Lot no. 202011033), 15 g Poria cocos (Schw.) Wolf. (Lot no. 201100091), 15 g Scutellaria barbata D. Don. (Lot no. 200702711), 15 g Hedyotis diffusa Willd (Lot no. 201100751), 10 g Bupleurum chinense DC. (Lot no. 200901861), 10 g Paeonia lactiflora Pall. (Lot no. 201200049), and 5 g Glycyrrhizae Radix Et Rhizoma Praeparata Cum Melle (Lot no. 2011208) purchased from the Fourth Clinical Medical College of Guangzhou University of Chinese Medicine were soaked in 1000 ml distilled water for 30 min and then were decocted for 30 min. The extraction procedure was repeated twice. The extracts were pooled and the supernatant was collected by filtration. Then, the supernatant was lyophilized in the vacuum freeze-drying machine (ALPHA2-4/LSC, Martin Christ, Germany) to prepare dried powder. The dried powder was redissolved in DMEM (Gibco, USA) complete culture medium to 100 mg/ml and filtered with a 0.22 *μ*m pore size filter and stored at -20°C for further use.

Based on network pharmacology results and previous research from our research team [8], the main ingredients (gallic acid, luteolin, quercetin, kaempferol, baicalein, and wogonin) of YQJPJD formula were analyzed by HPLC-Q-TOF-MS/MS (1290-6540 series, Agilent Technology, USA), and an ACQUITY BEH C18 (2.1 × 150 mm, 1.7 *μ*m) column at 40°C was used for the analysis. The mobile phase consists of phase A (0.1% formic acid in water) and phase B (acetonitrile) with a flow rate of 0.2 ml/min. The standards, reagents, and instruments involved in composition identification are provided by the China National Analytical Center in Guangzhou.

#### 2.7.2. Cell Cultures and Cell Viability Measurements

Hep3B and HepG2 cells were gifted by Prof. George G. Chen (The Chinese University of Hong Kong, Hong Kong, China). These two cell lines were cultured in DMEM complete culture medium with 10% fetal bovine serum (FBS; Gibco, USA) and 1% penicillin/streptomycin (Gibco, USA). Hep3B or HepG2 cell lines seeded into 96-well plates at a density of 4 × 10^3^ cells/well were treated with various concentrations (0, 0.5, 1, 1.5, 2, 2.5, 3, 3.5, and 4 mg/ml) of YQJPJD formula for 24, 48, and 72 hours, respectively. Subsequently, cells (in each well) were incubated with 10 *μ*l of MTT (5 mg/ml; Solarbio, China), and then, cells were cultured at 37°C for another 4 h. Afterwards, the supernatants were discarded and 100 *μ*l of dimethyl-sulfoxide (DMSO; Sigma, USA) was added to each well. The absorbance was measured at 490 nm using a microplate reader (168-1130A, Bio-Rad, USA).

#### 2.7.3. Apoptosis Assay and Hoechst 33342 Staining

According to the result of MTT assay, the dosages of 1, 2, and 3 mg/ml were selected for the following studies in vitro. Hep3B or HepG2 cell lines seeded into 6-well plates at a density of 1 × 10^6^ cells/well were treated with different concentrations (0, 1, 2, and 3 mg/ml) of YQJPJD formula for 48 h. Apoptosis assay was utilized to assess apoptosis of HepG2 and Hep3B cells using the Annexin V-FITC/PI Apoptosis Detection Kit (Beyotime, China) according to the manufacturer's protocol. Briefly, HepG2 or Hep3B cells were collected by centrifugation (1000 rpm for 3 min), washed with precooled PBS (Gibco, USA), stained with Annexin V-FITC and propidium iodide, and quantified by flow cytometry (Beckman Coulter, USA). Also, apoptotic condensed nuclear changes were identified using Hoechst 33342 (Beyotime, China) staining according to the manufacturer's instructions.

#### 2.7.4. Wound Healing Assay

The scratch wound healing assay was utilized to measure cell migratory ability. Hep3B or HepG2 cells were seeded in 12-well plates (5 × 10^5^/well) and were cultured overnight. Then, a 200 *μ*l sterile pipette tip was used to make linear scratch wounds. The cells were then treated with various concentrations (0, 1, 2, and 3 mg/ml) of YQJPJD formula, and photomicrographs (×100) were captured at 0 h and 48 h using the inverted fluorescence microscope (DMi8, Leica, Germany). The area of each scratch wound was determined by ImageJ software (https://imagej.net/software/imagej/). Wound healing rate = (0 h scratch area − 48 h scratch area)/0 h scratch area × 100%.

#### 2.7.5. Transwell Migration and Invasion Assays

The migration and invasion capacities of Hep3B and HepG2 cells were measured with a 24-well transwell plate (Corning, USA). In transwell migration assay, Hep3B or HepG2 cells were seeded in the upper chamber (5 × 10^4^/250ul/well) and were treated with various concentrations (0, 1, 2, and 3 mg/ml) of YQJPJD formula, and the lower chamber was added with 750 *μ*l DMEM medium containing 20% FBS. Cells were incubated for 48 h (37°C, 5% CO_2_), and then, cells were fixed with 75% ethanol for 30 min and stained with 0.1% crystal violet (Aladdin, China) for 15 min. The migrated cells were photographed under a microscope in 3 randomly selected fields by using Evos XL Core microscope (Life Technologies), and cell number was counted with ImageJ. For the transwell invasion assay, Matrigel (Cultrex; Trevigen Inc., USA) was diluted and placed in the upper chamber, and the following steps were the same as those mentioned above in transwell migration assay.

#### 2.7.6. Quantitative Real-Time PCR (qRT-PCR)

Hep3B or HepG2 cell lines seeded into 6-well plates at a density of 1 × 10^6^ cells/well were treated with various concentrations (0, 1, 2, and 3 mg/ml) of YQJPJD formula for 48 h. Total RNA was extracted using RNAiso Plus reagent (Takara, Japan) according to the manufacturer's instructions. Concentration of the extracted RNA was measured by NanoDrop Spectrophotometer (Thermo, USA), cDNA was generated from total RNA by reverse transcription using the PrimeScript RT Master Mix (Takara, Japan), and the qRT-PCR was performed using TB Green® Premix Ex Taq™ (Takara, Japan) in the CFX Connect Real-Time System (Bio-Rad, USA). The PCR reaction conditions were conducted as follows: predenaturation at 95°C for 120 sec followed by 40 cycles of 95°C for 10 sec, 60°C for 30 sec, and 72°C for 20 sec. The fold change for target genes normalized by internal control (*β*-actin) was determined by 2^−*ΔΔ*CT^ method. The following primers were used: *β*-actin forward 5′-AGGATGCAGAAGGAGATCAC-3′ and reverse 5′-TGTAACGCAACTAAGTCATAG-3′; *β*-catenin forward 5′-CATCTACACAGTTTGATGCTGCT-3′ and reverse 5′-GCAGTTTTGTCAGTTCAGGGA-3′; MAPK3 forward 5′-CTACACGCAGTTGCAGTACAT-3′ and reverse 5′-CAGCAGGATCTGGATCTCCC-3′; ROHA forward 5′-GGAAAGCAGGTAGAGTTGGCT-3′ and reverse 5′-GGCTGTCGATGGAAAAACACAT-3′; and RAC1 forward 5′-ATGTCCGTGCAAAGTGGTATC-3′ and 5′-CTCGGATCGCTTCGTCAAACA-3′.

#### 2.7.7. Western Blot Analysis

Western blot was performed with reference to our previous study [8]. Total protein was extracted from the cells into the RIPA lysis buffer containing protease inhibitor (Zhonghuihecai, China). Protein lysates were then resolved in SDS-PAGE (Beyotime, China) gel and transferred to polyvinylidene fluoride (PVDF) membrane (Merck Millipore). The PVDF membranes were probed with primary antibodies: PI3K, p-PI3K, Akt, p-Akt (Cell Signaling Technology, USA), and *β*-actin (Santa Cruz, USA). A 1 : 2000 dilution of the m-IgG*κ* BP-HRP and mouse anti-rabbit IgG-HRP (Santa Cruz, USA) was used as the secondary antibody. The results were visualized with the ChemiDoc Touch (Bio-Rad, USA), and ImageJ was used for protein level quantification. Expression levels of the proteins were normalized with *β*-actin; then, the treatment group was normalized with the control group.

#### 2.7.8. Statistical Analysis

Experimental data in this study were expressed with mean ± standard deviation (SD). Statistical analyses were completed using SPSS version 22.0. Differences between groups were performed by one-way analysis of variance (ANOVA) test followed by the Bonferroni analysis when the variances were homogeneous, and Welch's ANOVA and Dunnett's T3 tests were performed when the variances were irregular. The difference was considered statistically significant for *p* < 0.05. Statistical graphs were plotted by GraphPad Prism version 8.

## 3. Results

### 3.1. Bioactive Ingredients and Targets of YQJPJD Formula

The number of bioactive ingredients of each Chinese materia medica in the five databases is summarized in Table 1. After the removal of duplications, a total of 164 bioactive ingredients were obtained, and 1506 corresponding targets were identified. Besides, we obtained 936, 578, 74, and 115 HCC-related target genes from MalaCards, SymMap, TCMIP, and HERB databases, respectively, and a total of 963 potential therapeutic targets for HCC were identified after excluding duplicates.

### 3.2. Network of YQJPJD Formula Bioactive Ingredients and Common Targets

As shown in Figure 1, the Venn diagram exhibited the intersection (common targets) of YQJPJD formula and HCC, and a total of 224 common targets were determined. In this study, the 224 common targets are considered to be the targets for YQJPJD formula to exert its anti-HCC effect. In order to study the interaction between bioactive ingredients of YQJPJD formula and common targets, a network was constructed by using Cytoscape (Figure 2). As displayed in Figure 2, the network of YQJPJD formula bioactive ingredients and common targets included 369 nodes (145 bioactive ingredients and 224 target genes) and 1985edges, and the ten Chinese materia medicas were classified into three types (“replenishing qi and strengthening spleen,” “clearing heat and removing toxicity,” and “dispersing stagnated liver qi and nourishing blood”). Also, the bioactive ingredients connected with the most common targets (count ≥ 20) in the network are shown in Table 2, and quercetin, wogonin, luteolin, baicalein, etc. might be the important ingredients of YQJPJD formula against HCC.

### 3.3. Results of PPI and Hub Gene Analyses

A PPI network with 212 nodes (proteins of common targets) and 1457 edges (interaction relationships) was constructed using STRING database, and this result was visualized by Cytoscape (Figure 3(a)). In Figure 3(a), the larger the node or the darker the node color, the greater the degree value, indicating that the node was connected with more common targets in the PPI network. Then, based on the degree value, the top 15 nodes were selected as hub genes, including TP53, AKT1, STAT3, MAPK1, MAPK3, SRC, JUN, PIK3CA, PIK3R1, HRAS, MAPK8, EGFR, KRAS, RHOA, and RAC1 (Figure 3(b)).

### 3.4. The Results of KEGG and GO Analyses

The results of GO analysis demonstrated that the common targets of YQJPJD formula and HCC were mainly enriched in BP items such as negative regulation of apoptotic process, positive regulation of transcription DNA-templated, positive regulation of gene expression, response to drug, and regulation of cell proliferation; CC items such as cytosol, nucleus, cytoplasm, and nucleoplasm; and MF items such as enzyme binding, transcription factor binding, protein binding, and identical protein binding (Figure 4). Moreover, the result of KEGG analysis displayed that common targets were associated with pathways in cancer, hepatitis B, proteoglycans in cancer, PI3K-Akt, Ras, FoxO, Rap1 pathway, etc., and the first 20 signaling pathways are shown in Figure 5. In Figure 5, the bubble chart on the right showed the top 20 KEGG pathways based on gene count, and the Sankey diagram on the left showed the 15 hub genes participating in the top 20KEGG.

### 3.5. Results of Expression and Survival Analyses of Hub Genes

After screening hub genes, the mRNA expression levels of hub genes in HCC were analyzed by UALCAN database. The result of UALCAN showed that the mRNA expression levels of TP53, AKT1, MAPK1, MAPK3, SRC, PIK3CA, HRAS, MAPK8, KRAS, RHOA, and RAC1 in HCC samples were significantly higher than that in normal liver tissues, the mRNA expression of JUN in HCC was lower than that in normal liver tissue, and there was no significant difference in the mRNA expression of STAT3, EGFR, and PIK3R1 (Figure 6).

Through the HPA database, the representative images of immunohistochemistry staining for 15 hub genes in HCC and normal liver tissues were obtained, and the results are shown in Figure 7. The protein expression levels of TP53, MAPK1, MAPK3, PIK3CA, MAPK8, RHOA, and RAC1 in HCC were higher than that in normal liver tissue, while the expression of STAT3, HRAS, and KRAS protein was lower in HCC. The protein expression levels of AKT1 and EGFR were lower in normal liver tissue and HCC, and PI3KR1, SRC, and JUN were not detected in HCC.

The results of the survival analysis of 15 hub genes are shown in Figure 8. KM survival curves exhibited that the high mRNA expression levels of TP53, STAT3, PIK3R, and EGFR were related to longer OS in HCC patients, while the high expression levels of MAPK3, SRC, HRAS, RHOA, and RAC1 were associated with shorter OS. Besides, there was no statistical difference in other hub genes.

### 3.6. Molecular Docking Result

Based on the network of YQJPJD formula bioactive ingredients and common targets, the hub genes, whose mRNA expression was consistent with the protein expression and survival analysis was statistically significant, were selected for molecular docking. In this study, we selected the protein receptors of MAPK3, RAC1, and RHOA to dock with their corresponding bioactive ingredients. The results of molecular docking were evaluated by affinity values from AutoDock Vina program. When the affinity value is less than -5.0 kcal/mol, it is considered that the bioactive ingredient had a good binding affinity with the protein receptor. As displayed in Table 3 and Figure 9, the bioactive ingredients of YQJPJD formula bound well to the protein receptors of MAPK3, RAC1, and RHOA.

### 3.7. Results of HPLC-Q-TOF-MS/MS and MTT Assay

According to the results of network pharmacology and previous research [8], HPLC-Q-TOF-MS/MS was used to detect whether the YQJPJD formula contained gallic acid, luteolin, quercetin, kaempferol, baicalein, and wogonin, and the result is shown in Figure 10 and Table 4. The effect of YQJPJD formula on the proliferation and growth of HepG2 and Hep3B cells was detected by MTT assay (24 h, 48 h, and 72 h). The results of MTT experiment showed that different concentrations of YQJPJD formula had an inhibitory effect on Hep3B and HepG2 cells. In a certain concentration range, the cell viability of Hep3B and HepG2 cells decreased gradually with the increase of drug concentration and exposure time. Thus, YQJPJD formula could inhibit the proliferation of Hep3B and HepG2 cells in a time- and concentration-dependent manner (Figure 11).

### 3.8. Effect of YQJPJD Formula on Apoptosis in Hep3B and HepG2 Cells

Based on the experimental results of MTT assay, YQJPJD formula with the concentration of 0 mg/ml (control group), 1 mg/ml, 2 mg/ml, and 3 mg/ml and the 48 h time point were selected for further experiments. As displayed in Figure 12(a), the total apoptotic rate of Hep3B cells increased at 48 h with the increase of the concentration of YQJPJD formula, and the difference was statistically significant; although there was no statistically significant difference in HepG2, apoptotic rate tended to increase from 2 mg/ml. Besides, Hoechst 33342 was utilized to detect the morphological changes of apoptotic cells. Due to the structural changes of DNA and the increase of cell membrane permeability of apoptotic cells, Hoechst 33342 could easily enter apoptotic cells to bind to DNA, and the blue fluorescence intensity of apoptotic cells was higher than that of normal cells. As shown in Figure 12(b), Hep3B and HepG2 cells showed typical apoptosis characters with YQJPJD formula treatment for 48 h.

### 3.9. Effect of YQJPJD Formula on Migration and Invasion of Hep3B and HepG2 Cells

Firstly, the migration activity of Hep3B and HepG2 cells was measured by the scratch wound healing assay. The result showed that wound healing area in HepG2 and Hep3B cells increased following treatment with YQJPJD formula, and wound healing rate decreased with the increase of YQJPJD formula concentration in a dose-dependent manner (Figure 13). Then, cell migration was also determined by transwell migration assay, and the result indicated that YQJPJD formula (2 mg/ml and 3 mg/ml) could significantly inhibit migration capacity of Hep3B and HepG2 cells compared to the control group (0 mg/ml) (Figure 14(a)). Moreover, the result of transwell invasion assay demonstrated that the number of invading Hep3B or HepG2 cells was decreased following treatment with YQJPJD formula compared with the control group (Figure 14(b)).

### 3.10. Effect of YQJPJD Formula on the mRNA Expression of *β*-Catenin, MAPK3, RAC1, and RHOA

Based on the findings of network pharmacology, bioinformatic analysis, and the literature report [23], we detected the mRNA expression levels of *β*-catenin, MAPK3, RAC1, and RHOA in Hep3B and HepG2 cells after treatment with YQJPJD formula for 48 hours (Figure 15). The result of qRT-PCR displayed that in Hep3B and HepG2 cells, the mRNA expression of *β*-catenin in YQJPJD formula group was significantly lower than that in the control group. In HepG2 cells, the mRNA expression of MAPK3 in YQJPJD formula group (1 mg/ml and 3 mg/ml) was remarkably lower than that in the control group, and the mRNA expression of RHOA in YQJPJD formula group (3 mg/ml) was significantly lower than that in the control group (Figure 15(a)). Besides, the difference in MAPK3, RAC1, and RHOA of Hep3B cells did not reach statistical significance; although the mRNA level of RAC1 in YQJPJD formula group did not reach statistical difference, it had a decreasing trend (Figure 15(b)).

### 3.11. Effect of YQJPJD Formula on the Expression of PI3K/Akt Pathway-Related Proteins

On the basis of network pharmacology, the changes in protein expression of total PI3K, total Akt, phosphorylated-PI3K (p-PI3K), and phosphorylated-Akt (p-Akt) were detected by the western blot method to clarify the regulatory effect of YQJPJD formula on PI3K/Akt pathway. The results showed that the protein expression levels of p-PI3K and p-Akt were downregulated in HepG2 after treatment with YQJPJD formula (3 mg/ml) compared with the control group (Figure 16(a)), and the protein expression levels of total Akt, p-PI3K, and p-Akt also decreased in Hep3B after treatment with YQJPJD formula (3 mg/ml) compared with the control group (Figure 16(b)). Thus, YQJPJD formula could inactivate the phosphorylation of both PI3K and Akt in HCC cells.

## 4. Discussion

YQJPJD formula is a TCM prescription for the treatment of HCC, which is composed of 10 kinds of Chinese materia medicas, such as *Phyllanthus urinaria L.* and *Astragalus membranaceus (Fisch.) Bunge*. It is generally believed that the TCM pathogenesis of HCC lies in “Yu” (stasis of blood or qi), “Du” (toxicity), and “Xu” (deficiency), and “spleen (a concept of a comprehensive functional unit which is mainly involved in the digestive system and immune system) deficiency” occupies an important position in TCM pathogenesis of HCC. Also, the TCM treatment principles include “Qingre Jiedu” (clearing heat and removing toxicity) and “Jianpi Liqi” (tonifying spleen and regulating qi) [24, 25]. According to the TCM theory, YQJPJD formula is a representative prescription for “Yiqi Jianpi Jiedu” (replenishing qi, strengthening spleen, and removing toxicity), which is in line with the TCM pathogenesis of HCC [9]. In this study, a variety of valuable bioactive ingredients and corresponding targets of YQJPJD formula were found through network pharmacology, which have the potential to be further developed for treating HCC. Network of YQJPJD formula bioactive ingredients and common targets summarized several significant ingredients (e.g., quercetin, wogonin, luteolin, baicalein, stigmasterone, 24-ethylcholest-4-en-3-one, calycosin, kaempferol, ellagic acid, and beta-sitosterol) that may play a therapeutic role. Quercetin, a bioactive flavonoid, has been reported to have a direct anti-HCC effect and inhibit Akt/mTOR pathway [26]. Wogonin could suppress the activity of MMP-9 and inhibit migration and invasion in HCC [27]. Luteolin and kaempferol could induce apoptosis by increasing the activity of caspase-3 and would not be harmful to normal hepatocytes, which were thought to be used as anti-HCC drugs [28]. In addition, calycosin could produce an anti-HCC effect by activating ROS-mediated MAPK and STAT3 pathways [29]. It was reported that *β*-sitosterol and baicalein can induce apoptosis of HCC cells by regulating apoptosis-related genes [30, 31]. Zhong et al. [32] found that ellagic acid synergistically enhanced the inhibitory effect of doxorubicin and cisplatin on HCC. Overall, the ingredients of YQJPJD formula are complicated and diversified, and many of them have strong anti-HCC activity. Besides, several ingredients, such as stigmasterone and 24-ethylcholest-4-en-3-one, have not been reported in HCC yet, which brings some inspiration to future research.

The results of GO analysis demonstrated that the common target genes of YQJPJD formula and HCC were significantly involved in the cellular components and biological processes associated with gene regulation and cell proliferation, and the molecular function may be related to physiological metabolism in the liver. KEGG analysis showed that YQJPJD formula may play an anti-HCC effect through the pathways related to malignant tumors. HBV genome can be integrated into the host genome to cause carcinogenesis, and chronic hepatitis B-related inflammation can lead to the accumulation of HCC-related genetic and epigenetic defects [33]. It has been reported that PI3K/Akt was associated with poor survival, tumor metastasis, and vascular invasion in patients with HCC, which may be the key to HCC drug development [34]. Moreover, factors that are negatively regulated downstream of PI3K/Akt pathway are forkhead box O family (FOXO) members, and evidence suggests that FOXOs, especially FOXO3, are related to tumorigenesis [35]. CD73 could promote the progression and metastasis of HCC via activating PI3K/Akt pathway by inducing Rap1-mediated membrane localization of P110*β* [36]. Proteoglycans, the extracellular matrix components of liver microenvironment, were reported to play an important role in the development of HCC and have the potential to become therapeutic targets for HCC [37]. In addition, the activation of RAS/MAPK pathway and the dysregulation of microRNA are correlated with the occurrence and development of HCC. Therefore, YQJPJD formula may play an anti-HCC effect by regulating tumorigenesis-related pathways.

Based on PPI analysis, we found that 15 hub genes may be the targets for YQJPJD formula to play an anti-HCC effect. Among them, the mRNA expression of 12 hub genes was differentially expressed in HCC and normal liver tissues, and the protein expression of 7 hub genes (TP53, MAPK1, MAPK3, PIK3CA, MAPK8, RHOA, and RAC1) was consistent with that of mRNA. Additionally, among the 7 hub genes whose protein expression was consistent with the expression pattern of mRNA, we found that the mRNA expressions of 3 hub genes (MAPK3, RHOA, and RAC1) were correlated with poor OS. The results of molecular docking displayed that MAPK3, RHOA, and RAC1 had a good affinity with the corresponding ingredients in YQJPJD formula, and Van der Waals forces, alkyl, hydrogen bonds, and Pi-Pi stacking were involved in the interactions between receptors and ingredients. As reported in the literature, HCC patients with hyperphosphorylated mitogen-activated protein kinase (MAPK3/ERK1) had a high recurrence rate and a relatively short OS time [38]. Rac Family Small GTPase 1 (RAC1) is a regulator of several cell processes, such as cell cycle, intercellular adhesion, movement, and epithelial differentiation, and functions as a tumor oncogene in HCC [39]. RHOA (member of RAS homologous gene family A) is generally overexpressed in HCC, and its expression is associated with poor prognosis [40]. Therefore, previous studies have made our results more convincing. Also, there are few reports about target genes found in network pharmacology, which would provide new references for anti-HCC new drug development basis. As the target genes that may be obtained by different screening methods are different, and the massive information of each database is constantly updated, the results of network pharmacology may not fully reflect all the key target genes of YQJPJD formula in the treatment of HCC, which needs further study in the future.

In the experimental section, it was confirmed that gallic acid, quercetin, luteolin, kaempferol, baicalein, and wogonin occurred in YQJPJD formula by using HPLC-Q-TOF-MS/MS. The MTT assay revealed that YQJPJD formula could inhibit the proliferation of HepG2 and Hep3B cells in a dose- and time-dependent manner, and the lower concentration of YQJPJD formula (such as 0.5 mg/ml) has a more obvious inhibitory effect on Hep3B than that of HepG2 cells. Compared with the control group, YQJPJD formula could significantly promote the apoptosis of Hep3B cells, and apoptotic rate increased with increasing drug concentrations. The result of apoptosis assay showed that HBV-related HCC may be more sensitive to YQJPJD formula. Additionally, the scratch wound healing and transwell assays showed that YQJPJD formula could also suppress the migration and invasive abilities of HCC cells. Thus, the experimental results revealed that YQJPJD formula, which has the TCM effect of “Yiqi Jianpi” (replenishing qi and strengthening spleen) and “Jiedu” (removing toxicity), could suppress HCC cell proliferation, migration, and invasion and promote cell apoptosis. Previous studies have also shown that TCM prescriptions with the TCM effect of “strengthening spleen” (Jianpi in Chinese) or “removing toxicity” (Jiedu in Chinese) could inhibit the proliferation, migration, and invasion of HCC cells and regulate the signal transduction pathway [41, 42].

In order to further explore the possible mechanism of YQJPJD formula in the treatment of HCC, several target genes and pathways predicted in network pharmacology were verified. The result of qRT-PCR experiment demonstrated that YQJPJD formula could inhibit the mRNA expression of *β*-catenin in both Hep3B and HepG2 cells, as well as the MAPK3 and RHOA in HepG2. Research reported that about one-third of patients with HCC showed gain-of-function mutations of *β*-catenin that correlate with poor T cell infiltrates and unresponsiveness to immunotherapy with checkpoint inhibitors [23]. The result of qRT-PCR also revealed that there were differences in the mechanism of YQJPJD formula in the treatment of HBV-related HCC and nonviral HCC. Moreover, the results of western blot displayed that a higher concentration of YQJPJD formula could remarkably reduce the protein expression levels of p-PI3K and p-Akt in HepG2 and Hep3B cells, indicating that YQJPJD formula may influence the proliferation, apoptosis, migration, and invasion of HCC cells by inhibiting the activation of PI3K/Akt pathway. Previous research indicated that the activation of PI3K/Akt pathway leads to HCC cell proliferation, migration, invasion, and cell cycle arrest but suppresses cell apoptosis [43]. RHOA could increase the activity of the PI3K/Akt pathway and reduces production of chemokines related to effector T cell recruitment [44]. In the Wnt/*β*-catenin pathway, glycogen synthase-3*β* (GSK-3*β*) can phosphorylate *β*-catenin, resulting in ubiquitin degradation of *β*-catenin. This process can be reversed by Akt-induced phosphorylation of GSK-3*β*, resulting in the accumulation of *β*-catenin, thus inducing the growth and metastasis of cancer cells [45]. There are some shortcomings of experimental section in our research. Firstly, no associated agonists and inhibitors were used in the in vitro experiment. Furthermore, our study lacks the verification of animal experiment. These limitations demonstrated the need for future research.

## 5. Conclusions

Overall, YQJPJD formula, a representative prescription for “Yiqi Jianpi Jiedu” (replenishing qi, strengthening spleen, and removing toxicity), has the characteristics of multicomponent, multitarget, and multipathway for the treatment of HCC. Moreover, YQJPJD formula may inhibit the proliferation, migration, and invasion, as well as promote the apoptosis of HCC cells by regulating MAPK3, RHOA, *β*-catenin, and PI3K/Akt signaling pathway.

## Figures and Tables

**Figure 1:** Venn diagram of YQJPJD formula targets and HCC targets.

**Figure 2:** The network of YQJPJD formula bioactive ingredients and common targets. The green, yellow, and purple nodes represent Chinese materia medicas for “replenishing qi and strengthening spleen,” “clearing heat and removing toxicity,” and “dispersing stagnated liver qi and nourishing blood,” respectively. The blue diamond nodes stand for the common targets of YQJPJD formula and HCC. In the green nodes, V, triangle, circle, hexagon, and rectangle represent the bioactive ingredients of *Astragalus membranaceus (Fisch.) Bunge* (Huangqi in Chinese), *Codonopsis pilosula (Franch.) Nannf.* (Dangshen in Chinese), *Atractylodes macrocephala Koidz.* (Baizhu in Chinese), *Poria cocos (Schw.) Wolf.* (Fuling in Chinese), and *Glycyrrhizae Radix Et Rhizoma Praeparata Cum Melle* (Zhigancao in Chinese), respectively. In the yellow nodes, rectangle and circle represent the bioactive ingredients of *Scutellaria barbata D. Don.* (Banzhilian in Chinese) and *Hedyotis diffusa Willd* (Baihuasheshecao in Chinese), respectively. In the purple nodes, circle and rectangle represent the bioactive ingredients of *Bupleurum chinense DC.* (Chaihu in Chinese) and *Paeonia lactiflora Pall.* (Baishao in Chinese), respectively. The red rectangle represents the common ingredients of multiple Chinese materia medicas, including *Phyllanthus urinaria L.* (Yexiazhu in Chinese).

**Figure 3:** The PPI network of common targets and hub genes. (a) The PPI network of common targets includes 212 nodes and 1457 edges. (b) The network of 15 hub genes.

**Figure 4:** Top 10 most significant items in each category in GO analysis. FDR: false discovery rate; BP: biological process; CC: cellular component; MF: molecular function.

**Figure 5:** KEGG pathway enrichment analysis of common targets (the first 20 pathways with target count ≥ 10 and FDR < 0.05). FDR: false discovery rate.

**Figure 6:** The mRNA expression levels of 15 hub genes in HCC. Expression levels of TP53 (a), AKT (b), STAT3 (c), MAPK1 (d), MAPK3 (e), SRC (f), JUN (g), PIK3CA (h), PIK3R1 (i), HRAS (j), MAPK8 (k), EGFR (l), KRAS (m), RHOA (n), and RAC1 (o) in HCC versus normal tissue (red: HCC; blue: normal).

**Figure 7:** The protein expression of 15 hub genes in HCC. The protein expression of TP53 (a), AKT (b), STAT3 (c), MAPK1 (d), MAPK3 (e), SRC (f), JUN (g), PIK3CA (h), PIK3R1 (i), HRAS (j), MAPK8 (k), EGFR (l), KRAS (m), RHOA (n), and RAC1 (o) in HCC and normal tissue.

**Figure 8:** Effect of the 15 hub genes on prognosis (overall survival time) in patients with HCC. KM survival curves of TP53 (a), AKT (b), STAT3 (c), MAPK1 (d), MAPK3 (e), SRC (f), JUN (g), PIK3CA (h), PIK3R1 (i), HRAS (j), MAPK8 (k), EGFR (l), KRAS (m), RHOA (n), and RAC1 (o).

**Figure 9:** Molecular docking result of YQJPJD formula bioactive ingredients and target proteins. The three-dimensional structures of protein receptors and bioactive ingredients were displayed in cartoon and gray bar forms, respectively. The interaction between the protein receptor and the bioactive ingredients of YQJPJD formula was shown in the two-dimensional diagram.

**Figure 10:** Analysis results of the bioactive ingredients of YQJPJD formula. (a) Total ion chromatograms were recorded in the negative (upper) and positive (lower) ionization modes for YQJPJD formula with an assigned identification of bioactive ingredients. (b) The structures of gallic acid, luteolin, quercetin, kaempferol, baicalein, and wogonin.

**Figure 11:** Effect of YQJPJD formula on the proliferation of HepG2 and Hep3B cells evaluated by MTT. Treatment with YQJPJD formula resulted in decreased cell viability/proliferation of HepG2 at 24 h (a), 48 h (b), and 72 h (c) ($\bar{x}\pm s$, *n* = 4). Treatment with YQJPJD formula resulted in decreased cell viability/proliferation of Hep3B at 24 h (d), 48 h (e), and 72 h (f) ($\bar{x}\pm s$, *n* = 4). ^∗^*p* < 0.05, ^∗∗^*p* < 0.01, and ^∗∗∗^*p* < 0.001 vs. 0 mg/ml (control).

**Figure 12:** Effect of YQJPJD formula on the apoptosis in HepG2 and Hep3B cells. (a) The total apoptosis rate of HepG2 (early apoptosis percentage+late apoptosis percentage) tended to increase in the 2 mg/ml and 3 mg/ml groups, but there were no statistically significant differences ($\bar{x}\pm s$, *n* = 3). YQJPJD formula (1, 2, and 3 mg/ml) increased the total apoptosis rate of Hep3B cells. (b) Morphologic changes of apoptotic cells (HepG2 and Hep3B) were assessed by Hoechst 33342 staining. In bar graphs, values are presented as mean ± SD. ^∗∗^*p* < 0.01 and ^∗∗∗^*p* < 0.001 vs. 0 mg/ml (control).

**Figure 13:** YQJPJD formula could inhibit the migration of HepG2 and Hep3B cells (wound healing assay). (a) The treatment with YQJPJD formula (1, 2, and 3 mg/ml) reduced wound healing rate compared with control (0 mg/ml), suggesting that it could suppress the migration ability of HepG2 cells (48 h). (b) The treatment with YQJPJD formula (2 and 3 mg/ml) reduced wound healing rate compared with control (0 mg/ml), indicating that it could inhibit the migration ability of Hep3B cells (48 h). In bar graphs, values are presented as mean ± SD. ^∗∗^*p* < 0.01 and ^∗∗∗^*p* < 0.001 vs. 0 mg/ml (control).

**Figure 14:** YQJPJD formula inhibited cell migration and invasion of HepG2 and Hep3B cells, which was determined by transwell assay (48 h). (a) YQJPJD formula remarkably suppresses cell migration in a concentration-dependent manner. (b) YQJPJD formula significantly inhibited cell invasion in a concentration-dependent manner. In bar graphs, values are presented as mean ± SD. ^∗^*p* < 0.05, ^∗∗^*p* < 0.01, and ^∗∗∗^*p* < 0.001 vs. 0 mg/ml (control).

**Figure 15:** The influences of YQJPJD formula on *β*-catenin, MAPK3, RAC1, and RHOA in HepG2 (a) and Hep3B (b) were examined by RT-qPCR (48 h). (a) YQJPJD formula treatment significantly inhibited *β*-catenin, MAPK3, and RHOA mRNA expressions of HepG2 compared with the control (0 mg/ml), and the difference in RAC1 did not reach statistical significance. (b) YQJPJD formula treatment significantly inhibited *β*-catenin mRNA expression of Hep3B compared with the control (0 mg/ml), and the difference in MAPK3, RAC1, and RHOA did not reach statistical significance. Values are presented as mean ± SD. ^∗^*p* < 0.05 and ^∗∗^*p* < 0.01 vs. 0 mg/ml (control).

**Figure 16:** Effect of YQJPJD formula on PI3K, p-PI3K, AKT, and p-Akt protein expression levels in HepG2 and Hep3B (48 h). (a) YQJPJD formula (3 mg/ml) treatment significantly inhibited p-PI3K and p-Akt protein expression levels of HepG2 compared with the control (0 mg/ml), and no significant differences in PI3K and Akt were observed. (b) YQJPJD formula treatment notably inhibited p-PI3K, Akt, and p-Akt protein expressions of Hep3B compared with the control (0 mg/ml), and no significant differences in PI3K were observed. Values are presented as mean ± SD. ^∗^*p* < 0.05 and ^∗∗^*p* < 0.01 vs. 0 mg/ml (control).

**Table 1:** The number of bioactive ingredients in each Chinese materia medica of YQJPJD formula.

Herb name	TCMSP	TCMIP	BATMAN-TCM	SymMap	HERB	Total
HQ	20	5	9	24	29	29
YXZ	—	—	2	—	3	3
DS	21	4	11	27	28	29
BZ	7	3	—	15	14	15
FL	15	8	5	22	24	24
BZL	29	5	5	27	35	35
BHSSC	7	—	1	8	8	8
CH	17	2	10	19	20	20
BS	13	7	9	27	29	29
ZGC	—	—	—	—	2	2

YXZ: *Phyllanthus urinaria L.*; HQ: *Astragalus membranaceus (Fisch.) Bunge*; DS: *Codonopsis pilosula (Franch.) Nannf.*; BZ: *Atractylodes macrocephala Koidz.*; FL: *Poria cocos (Schw.) Wolf.*; BZL: *Scutellaria barbata D. Don.*; BHSSC: *Hedyotis diffusa Willd*; CH: *Bupleurum chinense DC.*; BS: *Paeonia lactiflora Pall.*; ZGC: *Glycyrrhizae Radix Et Rhizoma Praeparata Cum Melle*.

**Table 2:** Data of bioactive ingredients of YQJPJD formula (common targets count ≥ 20).

Type	Component	Count	Herbs
Common ingredients	Quercetin	91	YXZ, HQ, BHSSC, BZL, CH
	Luteolin	55	DS, BZL
	Kaempferol	41	YXZ, HQ, CH, BS
	Beta-sitosterol	36	DS, BZ, BZL, BHSSC, CH, BS
	Stigmasterol	29	DS, BZL, BHSSC, CH
	Isorhamnetin	25	HQ, CH
	Sitosterol	24	DS, BZL, BS
	Baicalin	20	BZL, CH
	Formononetin	17	HQ BZ
	Spinasterol	13	DS, CH

Replenishing qi and strengthening spleen	Stigmasterone	44	DS
	Calycosin	43	HQ
	Ellagic acid	39	FL
	Beta-carotene	27	HQ
	Ellipticine	27	FL
	Poricoic acid C	25	FL
	*α*-Amyrin	22	BZ
	(+)-Medicarpin	21	HQ
	Astrapterocarpan	21	HQ
	DFV	21	ZGC

Clearing heat and removing toxicity	Wogonin	71	BZL
	Baicalein	47	BZL
	24-Ethylcholest-4-en-3-one	44	BZL
	Campesterol	26	BZL
	Clr	23	BZL

Dispersing stagnated liver qi and nourishing blood	(+)-Catechin	23	BS
	Areapillin	18	CH
	Pyrethrin II	18	BS
	Diosgenin	14	CH
	(-)-Catechin	13	BS

Count: common target count; YXZ: *Phyllanthus urinaria L.*; HQ: *Astragalus membranaceus (Fisch.) Bunge*; DS: *Codonopsis pilosula (Franch.) Nannf.*; BZ: *Atractylodes macrocephala Koidz.*; FL: *Poria cocos (Schw.) Wolf.*; BZL: *Scutellaria barbata D. Don.*; BHSSC: *Hedyotis diffusa Willd*; CH: *Bupleurum chinense DC.*; BS: *Paeonia lactiflora Pall.*; ZGC: *Glycyrrhizae Radix Et Rhizoma Praeparata Cum Melle*.

**Table 3:** Affinities of YQJPJD formula bioactive ingredients and target proteins.

No.	Target	Ingredient	Affinity (kcal/mol)
1	MAPK3	Quercetin	-9.2
2	MAPK3	Luteolin	-9.5
3	MAPK3	Baicalein	-9.3
4	RAC1	Wogonin	-6.9
5	RHOA	Wogonin	-8.1

**Table 4:** HPLC-Q-TOF-MS/MS data of the 6 ingredients from YQJPJD formula.

No.	tR (min)	m/z	Selected ion	Fragments (m/z)	Ingredient
1	3.375	169.0138	[M-H]-	169.0138, 125.0246, 79.0190	Gallic acid
2	20.915	285.0405	[M-H]-	285.0405, 241.0501, 199.0402, 175.0399, 133.0295, 107.0141, 61.9033	Luteolin
3	20.998	301.0354	[M-H]-	301.0354, 273.0394, 229.0490, 178.9983, 151.0037, 121.0296	Quercetin
4	23.545	285.0406	[M-H]-	285.0406, 211.0358, 151.0035	Kaempferol
5	24.128	269.0452	[M-H]-	269.0452, 197.0612	Baicalein
6	28.638	285.0754	[M+H]+	285.0754, 270.0529, 168.0554	Wogonin

## Data Availability

The data used and analyzed during the current study are available from the corresponding author on reasonable request.
